The article "Evaluation on Effect of Acupoint Application to Treat Idiopathic Edema of Perimenopausal Women Using the Segmentation Dictionary Learning Algorithm" was published in 2022. Journal: Comput Intell Neurosci.

# Evaluation on Effect of Acupoint Application to Treat Idiopathic Edema of Perimenopausal Women Using the Segmentation Dictionary Learning Algorithm

**DOI:** 10.1155/2022/2196782

**Published:** 2022-06-27

**Authors:** Jinfeng Li, Jiao Wang, Wenxia Zhao, Pei Wang, Min Li

**Affiliations:** Centre of Traditional Chinese Medical Science, Beijing Luhe Hospital Affiliated to Capital Medical University, Beijing 101149, China

## Abstract

This study aimed to explore the effect of ultrasound imaging in the diagnosis and evaluation of acupoint application in the treatment of idiopathic edema. In this study, an ultrasound imaging diagnosis based on the segmentation dictionary learning (S-DL) algorithm was proposed. In addition, the autoencoding algorithm (ASE) was compared with the traditional dictionary learning (DL) algorithm. The treatment effect, associated quantitative integral, and quality of life score of patients in two groups were compared. The results showed that the peak signal-to-noise ratio (PSNR), root mean square error (RMSE), and structural similarity (SSIM) of the S-DL algorithm were 32.45 dB, 0.654, and 0.0012, respectively, which were quite different compared to the ASE and DL algorithms, showing statistical significance (*P* < 0.05). As the noise level increased, the image reconstruction quality gradually decreased, but the S-DL algorithm obtained better image quality than the DL and ASE algorithms, and the difference was statistically great (*P* < 0.05). There was no significant difference in the average age and average course of the disease between the experimental group and the control group (*P* > 0.05). The overall treatment effect of patients in the experimental group was 96.77%, while that in the control group was 45.16%, and the difference between the two was statistically significant (*P* < 0.05). After treatment, the semiquantitative scores of fatigue, dizziness, palpitation, frequent urination, urgent urination, and dyspepsia of the experimental group were 1.18, 0.39, 0.72, 1.21, and 0.87, respectively, which were much lower than those of the control group statistically (*P* < 0.05). The score of quality of life of the experimental group of patients after treatment was 91.27 points, and that of the control group was 82.35 points, showing statistically great difference (*P* < 0.05). It showed that the algorithm performance of S-DL was relatively good, and the acupoint application therapy was better than traditional western medicine in the treatment of idiopathic edema, which reduces the discomfort of patients to a certain extent and improves the quality of life of patients.

## 1. Introduction

Idiopathic edema is also known as Mach syndrome. Idiopathic edema is more common in women aged 30–50 and is synonymous with terms such as periodic edema, obesity due to water and sodium retention, and idiopathic edema syndrome [1, 2]. Unlike cardiogenic, renal, hepatic, and other edema, idiopathic edema has no obvious cause. From a pathological point of view, it is caused by a disorder of water and salt metabolism and an abnormal increase in extracellular fluid in the subcutaneous space [3, 4]. The clinical symptoms of idiopathic edema can be expressed as follows: first is edema or edema of varying degrees after standing movement; second, most patients with idiopathic edema are obese, and their weight will also increase when edema occurs; third, some patients will have headaches due to intracranial edema, and when the edema disappears, the headaches will also be relieved. Fourth, a small number of patients will experience symptoms such as generalized pain and orthostatic hypotension after standing for a long time [5, 6]. In recent years, with the popularization of the concept of equality between men and women, women's social status has increased at the same time as their psychological pressure has increased, and the incidence of idiopathic edema has also increased year by year [7, 8]. Acupoint application is a common treatment method in traditional Chinese medicine therapy. It is to apply drugs on specific human acupoints through the dual action of drugs and acupoints, so as to achieve the purpose of treating and preventing diseases [4].

The article "Evaluation on Effect of Acupoint Application to Treat Idiopathic Edema of Perimenopausal Women Using the Segmentation Dictionary Learning Algorithm" was published in 2022. Journal: Comput Intell Neurosci.

Because the pathogenesis of idiopathic edema has not yet been cleared, and the clinical manifestations lack specificity, clinical diagnosis is difficult [9]. Ultrasound imaging is a commonly used clinical examination method, its operation is simple and fast, and there is no radiation damage, so it is popularized in clinical use [10]. However, the raw ultrasound data acquired by the ultrasound imaging map may form speckle noise and false texture due to the signal and equipment, resulting in unclear images. Doctors cannot obtain useful disease information from the original images in a timely and intuitive manner [11]. With the development of artificial intelligence, sparse representation theory has become a more popular direction in the research of image denoising. The theory is mainly divided into sparse decomposition reconstruction algorithm and dictionary design, but whether the image can be sparsely represented is determined by the dictionary learning algorithm [12]. For the choice of a dictionary, there are usually two methods. One is to select a fixed analysis dictionary, but it has limitations for the sparse representation of the sample, and it cannot guarantee the optimal sparse representation of the sample. The other is to train based on the existing sample data and learn the training samples to obtain an overcomplete dictionary library, such as MOD, K-SVD, and joint base dictionary [13, 14]. Therefore, a segmentation dictionary learning (S-DL) algorithm ultrasound imaging was proposed in this study, and it was applied to diagnose and evaluate the efficacy of acupoint application in the treatment of idiopathic edema.

The article "Evaluation on Effect of Acupoint Application to Treat Idiopathic Edema of Perimenopausal Women Using the Segmentation Dictionary Learning Algorithm" was published in 2022. Journal: Comput Intell Neurosci.

In summary, how to improve the efficacy of idiopathic edema is of great significance, and the DL algorithm has a better segmentation effect in the data processing of ultrasound imaging. Therefore, this study proposed ultrasound imaging based on S-DL algorithm, which was used in diagnosis and evaluation of the efficacy of acupoint application in the treatment of idiopathic edema. At the same time, autoencoding algorithm (ASE) and transmission DL algorithms were compared to provide effective data support for acupoint application treatment of idiopathic edema.

## 2. Materials and Methods

### 2.1. Research Objects and Their Grouping

In this study, 62 perimenopausal female patients admitted to the outpatient department from January 2020 to October 2021 were selected as the research objects. The patients were between 45 and 55 years old, with an average age of 49.34 ± 4.34 years old, and the course of the disease was 1 month to 2 years. All patients showed limb edema, and some patients were accompanied by facial edema. Relevant clinical data of the patients were collected, and the random number table method was adopted to randomly divide 62 patients into the experimental group and the control group, with each 31 patients. Patients in the experimental group received acupoint application treatment, and those in the control group received conventional treatment. This experimental study was approved and supported by the Medical Ethics Committee of hospital (2021-LHKY-001-02). All participants signed the written informed consent forms and volunteered to participate in this experimental study.

Inclusion criteria referring to the diagnostic criteria of idiopathic edema in Differential Diagnosis of Internal Medicine were as follows [15]: patients who were all perimenopausal women aged 45–55; patients whose weight difference between the morning and the evening was >1.4 kg; patients whose facial swelling was obvious in the morning, and the edema of the lower limbs was obvious in the afternoon, especially in the ankles and anterior tibia; and patients whose standing water test was positive. Exclusion criteria were as follows: patients whose edema was caused by organic diseases of the heart, liver, kidney, and other organs; patients whose edema was caused by nutritional deficiency; patients whose edema was caused by taking drugs (such as calcium channel blockers and receptor blockers); patients with serious immune diseases; and patients whose compliance was poor and unable to cooperate with the research.

The article "Evaluation on Effect of Acupoint Application to Treat Idiopathic Edema of Perimenopausal Women Using the Segmentation Dictionary Learning Algorithm" was published in 2022. Journal: Comput Intell Neurosci.

### 2.2. Treatment of Two Groups

In the experimental group, researchers determined the pathogenesis and syndrome types of the patient's edema based on traditional Chinese medicine (TCM) syndrome differentiation and treatment and then determined the acupoints and the required application of TCM based on the dialectical results. Acupoint selected included Xunshenjue, Zusanli, Fenglong, Liangqiu, Xuehai, and Diji. Prescription compositions included milk vetch 30 g, cinnamon sticks 15 g, aconite 10 g, sophora flavescens 15 g, aconite 10 g, angelica 15 g, safflower 15 g, long hair flower 15 g, star anise 15 g, pepper stem 10 g, sweet fragrant fruit 10 g, earthworm 10 g, mulberry 15 g, borneol 5 g, and Glauber's salt 30 g. The patient was instructed for external application of the medicine for 6 to 8 hours a day, ten days as a course of treatment, and two consecutive courses of treatment.

In the control group, the patients were instructed to take hydrochlorothiazide tablets (Xisen Pharmaceutical, H37021905) and spironolactone (Zhejiang Yatai Pharmaceutical Co., Ltd., H33020111) every day. Hydrochlorothiazide tablets were taken orally, once a day, and 25 mg once a day, and the Spironolactone was taken orally, once a day, and 20 mg once.

### 2.3. Imaging Examination

All patients were examined by the same ultrasound operator and the same instrument (Yumm MyLab Twice and Philips-iu22 color Doppler ultrasound): with the probe frequency of 5–12 MHz and high frequency variable frequency probe. The patient took the supine position and the prone position to fully expose the edema. After repeated scanning of the edema site, it should carefully observe the structural changes of the skin, subcutaneous tissue, deep fascia, and muscle tissue and measure the thickness. The imaging results were reviewed by two qualified doctors, and the comprehensive opinions of the two were taken after discussion with different opinions.

### 2.4. S-DL Algorithm

The S-DL algorithm extracted the main features from a large number of image blocks, so as to train a dictionary suitable for such image feature selection. The sparse representation means that only a few function bases in the complete dictionary, that is, a sparse atomic dictionary, can be used to represent the target object [16, 17]. It was supposed that the sample data set *M*=[*m*_1_, *m*_2_, *m*_3_ …, *m*_*y*_] ∈ *P*^*x*×*y*^ (*x* and *y* were the spatial dimensions of the sample), *K*={*k*_1_, *k*_2_, *k*_3_ …, *k*_*d*_} ∈ *P*^*x*×*d*^, and *x* < *d* (*d* was the number of function bases of the dictionary) and the constraint condition *k*_*d*_^*R*^*k*_*d*_ ≤ 1 were satisfied; then the linearity of the dictionary can be expressed as

(1) $$\begin{array}{c} \underset{\alpha }{\text{min}}{\left\|\alpha \right\|}_{0}s.t.m=K\alpha . \end{array}$$

In the above equation, ‖*α*‖_0_ represented the 0-th normal form and *α* was the sparse representation coefficient of *m*_*1*_.

The article "Evaluation on Effect of Acupoint Application to Treat Idiopathic Edema of Perimenopausal Women Using the Segmentation Dictionary Learning Algorithm" was published in 2022. Journal: Comput Intell Neurosci.

If *m* represented the image to be segmented, *K* represented the image block extracted from the image, *D* was the constructed dictionary, *α* represented the sparse representation coefficient, and *V* represented the set of *α*, then the objective function of the iterative optimization can be expressed as

(2) $$\begin{array}{c} \underset{K,D,V}{\min}\underset{pq}{\Sigma }{\left\|K_{pq}m-D\alpha_{pq}\right\|}_{2}^{2}+\nu {\left\|F_{u}m-n\right\|}_{2}^{2}, \end{array}$$

(3) $$\begin{array}{c} \text{s.t}{\left\|\alpha \right\|}_{0}\leq {\text{V}}_{0}\forall pq. \end{array}$$

In equations (2) and (3), *F*_*u*_ represented the Fourier transform and under-harvesting, *n* represented the k-space data obtained from under-harvesting, and *ν* represented the weight constant. The dictionary update uses the K-SVD [16] algorithm, and the sparse coefficient update uses the OMP [17] algorithm.

The basic idea of the K-means algorithm was to divide the data into K classes on the basis of minimizing the error function. The processing process of the algorithm was as follows. It should firstly specify the initial cluster center and the number of K initial clusters and then assign each data in the dataset to the nearest cluster center according to the proposed standard. If the data of the dataset *Y*={*x*_1_, *x*, *x*_3_ … …*x*_*i*_ … *x*_*n*_} was classified into K categories, the cluster center was ={*c*_1_, *c*_2_ …, *c*_*N*_ …, *c*_*K*_}. *d*_*iN*_(*x*_*i*_, *c*_*N*_) was to represent the distance between *x*_*i*_ and its corresponding cluster center *c*_*j*_, and the sum of the distances between all data points in the data set and the cluster center of their type was represented by the objective function H:

(4) $$\begin{array}{c} \begin{array}{c} H=\sum_{h=1}^{K}\sum_{i,i\epsilon c_{h}}d_{ih}\left(x_{i},c_{h}\right). \end{array} \end{array}$$

The smaller the objective function *H*, the more compact the clustering and the better the clustering quality. When selecting the Euclidean distance as the distance between the data *x*_*i*_ and its corresponding center *c*_*h*_, *x*_*i*_^*h*^ was the data sample belonging to cluster *h*, and *n*_*h*_ was the number of samples in cluster *h*:

(5) $$\begin{array}{c} H=\sum_{h=1}^{\text{K}}H_{n}=\sum_{h=1}^{K}\left[\sum_{i,i\epsilon c_{h}}{\left\|x_{i}^{h}-c_{h}\right\|}^{2}\right]. \end{array}$$

In order to minimize the objective function, each cluster center can be expressed as follows:

(6) $$\begin{array}{c} \begin{array}{c} c_{h}=\frac{1}{n_{j}}\sum_{i=1}^{n_{h}}x_{i}^{h}. \end{array} \end{array}$$

Figure 1 shows the processing result of the K-means clustering algorithm. It illustrated that the processed image had better clarity than the original image. The S-DL algorithm was to use the K-means clustering algorithm to cluster the images before the dictionary training of the images and use the segmented images to train the dictionary. The specific process is shown in Figure 2. The red marked area in the figure is stenosis and edema.

The article "Evaluation on Effect of Acupoint Application to Treat Idiopathic Edema of Perimenopausal Women Using the Segmentation Dictionary Learning Algorithm" was published in 2022. Journal: Comput Intell Neurosci.

### 2.5. Observation Indicators

The image quality mainly was evaluated with peak signal-to-noise ratio (PSNR), root mean square error (RMSE), and structural similarity index measurement (SSIM) to carry out various algorithms.

RMSE was a method of measuring the average error, which can evaluate the degree of data change. If $\hat{s}\left(q,r\right)$ was the target image, *s(q, r)* was the original image, *X* represented the pixel on the horizontal axis of the image, and *Y* represented the pixel on the vertical axis, then the calculation formula was as follows:

(7) $$\begin{array}{c} \text{RMSE}=\frac{1}{X\times Y}\overset{X}{\underset{q=1}{\sum }}\overset{Y}{\underset{r=1}{\sum }}{\left(\hat{s}\left(q,r\right)-s\left(q,r\right)\right)}^{2}. \end{array}$$

PSNR described the amount of noise in the image after noise reduction. Therefore, the higher the PSNR value, the less image noise, and the better the noise reduction effect.

(8) $$\begin{array}{c} \text{PSNR}=10{\text{log}}_{10}\frac{{\left(2^{n}-1\right)}^{2}}{\text{RMSE}}. \end{array}$$

Image similarity was mainly used to compare the SSIM of the content between two images. The similarity of the image content was judged according to the comparison result. The larger the SSIM value, the better the image quality evaluated. If *m* and *n* represented the original image and the image to be evaluated, the average value (*α*_*m*_, *α*_*n*_) was used to represent the brightness of the image, (*ρ*_*m*_, *ρ*_*n*_) was used to represent the contrast of the image, and *ρ*_*mn*_ was used to represent the structure of the image. The calculation equation was as follows:

(9) $$\begin{array}{c} \text{SSIM}\left(m,n\right)=\frac{\left(2\alpha_{m}\alpha_{n}+G_{1}\right)\left(2\rho_{mn}+G_{2}\right)}{\left(\alpha_{m}^{2}+\alpha_{n}^{2}+G_{1}\right)\left(\rho_{m}^{2}+\rho_{n}^{2}+G_{2}\right)}. \end{array}$$

It should observe the edema improvement effect of patients before and after treatment, and the effect evaluation standard is shown in Figure 3. At the same time, the accompanying symptoms such as fatigue, dizziness, panic, frequent urination, urgent urination, dyspepsia, and other emotional and physical discomfort changes of patients were observed and compared. Symptoms were represented by semiquantitative scores, as shown in Figure 4. The quality of life evaluation scale was used to evaluate the quality of life of patients before and after treatment. The quality of life assessment form was used to assess the quality of life of patients before and after treatment.

The article "Evaluation on Effect of Acupoint Application to Treat Idiopathic Edema of Perimenopausal Women Using the Segmentation Dictionary Learning Algorithm" was published in 2022. Journal: Comput Intell Neurosci.

Ineffective: edema and other symptoms and laboratory tests remain the same or repeated edema during treatment.

Improvement: edema and other symptoms are alleviated, and laboratory tests have improved.

Significantly effective: the edema has disappeared significantly, and the swelling and other symptoms of the whole body have basically disappeared.

Cure: the patient's edema and other symptoms disappeared, and urine output and weight returned to normal.

### 2.6. Statistical Analysis

SPSS2.0 software was used for data statistical analysis. The experimental data were expressed in terms of mean ± standard deviation ($\bar{\text{x}}$ ±*s*). After the normality and homogeneity of variance were tested, the measurement data conformed to the normal distribution. If the variances were uniform, the comparison between the two samples used the *t*-test, and the classification data comparison used the *χ*^2^ test. The I^2^ was adopted to assess the magnitude of heterogeneity. *P* < 0.05 indicated that there were significant differences in the data between the groups, which were statistically significant; otherwise, there was no difference without statistical significance.

## 3. Results

### 3.1. Comparison on Algorithm Performance

In this study, the self-encoding algorithm (SAE) and the traditional dictionary learning (DL) algorithm were introduced to compare with the S-DL algorithm adopted in this work. The results are shown in Figure 5. The peak signal-to-noise ratio (PSNR), structural similarity (SSIM), and mean square error (RMSE) of the S-DL algorithm were 32.45 dB, 0.654, and 0.0012, respectively, and compared with the SAE and DL algorithms, the differences were statistically significant (*P* < 0.05).

In order to further verify the effect of the algorithm on noise processing, the Gaussian distribution after adding complex noise was studied, the mean value was 0, and the variances were 0.5%, 1%, 3%, 5%, and 10% of the maximum value of the image domain, respectively. The central continuous acquisition of 15% was adopted to compare the PSNRs of the three algorithms, and the results are shown in Figure 6. As the noise level increased, the image reconstruction quality gradually decreased, but the S-DL algorithm obtained better image quality than the DL and ASE algorithms.

The article "Evaluation on Effect of Acupoint Application to Treat Idiopathic Edema of Perimenopausal Women Using the Segmentation Dictionary Learning Algorithm" was published in 2022. Journal: Comput Intell Neurosci.

Figure 7 shows an ultrasound imaging of a 47-year-old female patient with lower extremity edema. It shows that the echo and thickness of the patient's skin, subcutaneous tissue, and deep fascia were close to normal. However, the muscle layer tissue was thickened and the texture was thickened. In the muscles, there were lacunar-like nonechoic dark areas formed by fluid accumulation and tortuous and dilated small veins. The results of manual segmentation were compared with those of three algorithm segmentations, and the image quality of S-DL algorithm segmentation was the highest.

### 3.2. Statistical Analysis of the Age and Course

In order to verify the feasibility of this study, the age and course of the disease were compared between the experimental group and the control group. The results are shown in Figure 8. The average age of patients in the experimental group was 49.3 years and the average course of the disease was 13.1 months; the average age and average course of the disease of patients in the control group were 48.5 years and 12.3 months, respectively. The difference between the two was not obvious, and there was no statistical significance (*P* > 0.05).

### 3.3. Comparison on Treatment Effect

In this study, the treatment effects of the two groups of patients were compared through clinical manifestations and ultrasound examinations. The results are shown in Figure 9. In the experimental group, the numbers of cured, markedly effective, effective, and ineffective patients were 15 (48.38%), 11 (35.5%), 4 (12.9%), and 1 (3.22%), respectively, while those in the control group were 3 (9.7%), 5 (16.13%), 6 (19.35%), and 17 (54.82%), respectively. The total treatment effect of the experimental group was 96.77%, and that of the control group was 45.16%. The difference between the two was statistically significant (*P* < 0.05).

### 3.4. Changes of Semiquantitative Scores

In this study, the semiquantitative scores of the edema-associated symptoms of the two groups were measured and compared before and after treatment, and the results are shown in Figure 10. Before treatment, there was no significant difference in edema-associated symptoms (fatigue, dizziness, palpitation, frequent urination/urgent urination, and dyspepsia) between the two groups of patients, which was not statistically great (*P* > 0.05). After treatment, the fatigue, dizziness, palpitation, frequent urination/urgent urination, and dyspepsia semiquantitative scores of the experimental group were 1.18, 0.39, 0.72, 1.21, and 0.87, respectively, which were significantly lower than those of the control group (*P* < 0.05).

The article "Evaluation on Effect of Acupoint Application to Treat Idiopathic Edema of Perimenopausal Women Using the Segmentation Dictionary Learning Algorithm" was published in 2022. Journal: Comput Intell Neurosci.

### 3.5. Comparison on Score of Quality of Life between the Two Groups

The scores of quality of life between the two groups of patients were compared before and after treatment, and the results are shown in Figure 11. Before treatment, there was little difference between the scores of the experimental group and the control group, and it was not statistically significant (*P* > 0.05). After treatment, the average score of patients in the experimental group was 91.27 points, while the score of patients in the control group was 82.35 points, and the difference between the two was statistically significant (*P* < 0.05). At the same time, the scores of the experimental group and the control group after treatment were significantly different from the scores before treatment, but the difference between the experimental group and the patients was more obvious.

## 4. Discussion

Idiopathic edema is a syndrome caused by disorders of water and salt metabolism. Studies have shown that the disease is more common in middle-aged women, but the pathogenesis is not clear, and it is closely related to the increase in capillary permeability, the abnormal response of hormones to changes in body position, and diet [18–21]. Idiopathic edema is also called periodic edema, which often presents periodic attacks, which brings great troubles to patients' lives [22, 23]. As a result, this study proposed a S-DL algorithm, which was used in ultrasound imaging to diagnose and evaluate the efficacy of acupoint application in the treatment of idiopathic edema. In this study, the ASE algorithm was introduced and compared with the traditional DL algorithm and ASE algorithm in terms of PSNR, SSIM, and RMSE. The results showed that the PSNR, SSIM, and RMSE of the S-DL algorithm were 32.45 dB, 0.654, and 0.0012, respectively, which were greatly different from those of the ASE and DL algorithms statistically (*P* < 0.05). It indicated that the algorithm designed in this study showed better segmentation effect. In order to further verify the effect of the algorithm on noise processing, the Gaussian distribution after adding complex noise was studied, the mean value was 0, and the variances were 0.5%, 1%, 3%, 5%, and 10% of the maximum value of the image domain, respectively. The results showed that as the noise level increased, the image reconstruction quality gradually decreased, but the S-DL algorithm obtained better image quality than the DL and ASE algorithms, and the differences were statistically significant (*P* < 0.05). Such results were similar to the results of Tong et al. (2015) [24].

The article "Evaluation on Effect of Acupoint Application to Treat Idiopathic Edema of Perimenopausal Women Using the Segmentation Dictionary Learning Algorithm" was published in 2022. Journal: Comput Intell Neurosci.

In this study, the designed algorithm was applied to the clinical diagnosis and treatment of idiopathic edema patients. At the same time, the age and course of disease of the experimental group and the control group were compared to verify the feasibility of this study. The results showed that the average age of patients in the experimental group was 49.3 years and the average course of the disease was 13.1 months, while the average age of patients in the control group was 48.5 years and the average course of the disease was 12.3 months. There was no significant difference between the two (*P* > 0.05). In the experimental group, the proportions of cured, markedly effective, effective, and ineffective patients were 48.38%, 35.5%, 12.9%, and 3.22%, respectively, while those in the control group were 9.7%, 16.13%, 19.35%, and 54.82%, respectively. The total treatment effect of the experimental group was 96.77%, and that of the control group was 45.16%. The difference between the two was statistically significant (*P* < 0.05). The semiquantitative scores of the edema-associated symptoms of the two groups of patients before and after treatment were compared, and the results were similar to the study of Talukder et al. (2021) [25]. There was little difference between the two before treatment. After treatment, the semiquantitative scores of fatigue, dizziness, palpitation, frequent urination/urgent urination, and dyspepsia of the experimental group were 1.18, 0.39, 0.72, 1.21, and 0.87, respectively, which were much lower than those of the control group, and the difference was statistically significant (*P* < 0.05). Finally, the scores of quality of life between the two groups of patients before and after treatment showed that the scores of the experimental group and the control group were not significantly different before treatment, while the score in the experimental and control groups were 91.27 points and 82.35 points, respectively, showing statistically great difference (*P* < 0.05).

## 5. Conclusion

In order to explore the effect of ultrasound imaging in the diagnosis and evaluation of acupoint application in the treatment of idiopathic edema, this study proposed an ultrasound imaging diagnosis based on S-DL algorithm and compared ASE and DL algorithms to further verify the performance of S-DL algorithm. In addition, it compared the treatment effect, associated quantitative integral, and score of quality of life between the experimental group and the control group. It showed that the algorithm performance of S-DL was relatively good, and acupoint application therapy was better than traditional western medicine in the treatment of idiopathic edema, which reduces the discomfort of patients to a certain extent and improves the quality of life of patients. However, the current diagnosis of idiopathic edema lacked standardized syndrome differentiation criteria and efficacy judgment criteria, and there was also a lack of large-scale evidence-based medicine research. In general, the results of this study provided reliable data support for the diagnosis and treatment of idiopathic edema in clinical acupoint application.

The article "Evaluation on Effect of Acupoint Application to Treat Idiopathic Edema of Perimenopausal Women Using the Segmentation Dictionary Learning Algorithm" was published in 2022. Journal: Comput Intell Neurosci.

## Figures and Tables

**Figure 1:** BA image segmentation results with K-means clustering algorithm. (a) The original image; (b) the image processed by the K-means clustering algorithm.

**Figure 2:** The segmentation process of S-DL algorithm.

**Figure 3:** Effect evaluation criteria.

**Figure 4:** Semiquantitative scores standard.

**Figure 5:** Performance comparison of the three algorithms. A shows the comparison of the PSNR; B shows the comparison of SSIM; C shows the comparison of MSE. ^*∗*^Compared with S-DL algorithm, *P* < 0.05.

**Figure 6:** PSNR varied with noise. ^*∗*^Compared with DL algorithm, *P* < 0.05.

**Figure 7:** Comparison of segmentation results of three algorithms. (a) The image to be segmented; (b) the image after manual segmentation; (c) the image segmented by the SAE algorithm; (d) the image segmented by the DL algorithm; (e) the image segmented by the S-DL algorithm segmentation. The red marked area is the edema site.

**Figure 8:** Statistical analysis of age and disease course of the two groups of (a) and (b) showed the age and disease course information of the patients, respectively.

**Figure 9:** Comparison on treatment effect. ^*∗*^Compared with the experimental group, (*P*) < 0.05.

**Figure 10:** Comparison of integral values of two groups of patients. (a, b) The semiquantitative scores of edema accompanying symptoms before and after treatment, respectively. ^*∗*^Compared with the experimental group, *P* < 0.05.

**Figure 11:** Comparison on score of quality of life of patients. # and ^*∗*^indicate comparison on the score in the experimental group before and after the treatment, respectively. ^Δ^Compared with patients in the control group before treatment.

## Data Availability

The data used to support the findings of this study are available from the corresponding author upon request.
